The article "Effect of Entresto on Clinical Symptoms, Ventricular Remodeling, Rehabilitation, and Hospitalization Rate in Patients with Both Acute Myocardial Infarction and Acute Heart Failure" was retracted in 2023. Reasons: unreliable results or conclusions; concerns about the data; concerns about the peer review; concerns about the citations.

# Effect of Entresto on Clinical Symptoms, Ventricular Remodeling, Rehabilitation, and Hospitalization Rate in Patients with Both Acute Myocardial Infarction and Acute Heart Failure

**DOI:** 10.1155/2022/7650937

**Published:** 2022-08-16

**Authors:** Guiping Wang, Xiaokun Liu, Zimo Guo, Juanjuan Zhang, Shuping Zuo, Suya Sun, Yanan Zhao, Qi Zhang

**Affiliations:** ^1^Department of Cardiology, Tangshan Gongren Hospital, Tangshan, Hebei 063000, China; ^2^Department of Cardiology, Tangshan Gongren Hospital, North China University of Science and Technology, Tangshan, Hebei 063000, China

## Abstract

**Objective:**

To determine the influence of Entresto on clinical symptoms, ventricular remodeling (VR), and economic stress of patients with both acute myocardial infarction (AMI) and acute heart failure (AHF).

**Methods:**

Totally 120 patients with AMI complicated with AHF admitted to our hospital between January 2017 and August 2019 were enrolled and randomly assigned to an observation group (obs group) and a control group (con group) (each *n* = 60). The obs group was treated with Entresto, while the other with angiotensin-converting enzyme inhibitors (ACEI). After treatment, the efficacy on both groups was evaluated, and their cardiac function-associated indexes (left ventricular end-systolic diameter (LVESd), left ventricular end-diastolic dimension (LVEDd), left ventricular ejection fraction (LVEF), VR-associated indexes (interventricular septal thickness (IVST), and left ventricular mass index (LVMI)) were determined and compared before treatment and after 1 month of treatment. Additionally, their NT-pro-BNP, CRP, and TNF-*α* were tested and compared before and after treatment, and they were also compared in hospitalization time, treatment expense, readmission rate within one year after discharge, and adverse events.

**Results:**

After treatment, the obs group showed notably higher efficacy than the con group (*P* < 0.05). Before treatment, the two groups were not greatly different in LVESd, LVEDd, LVEF, IVST, LVMI, NT-pro BNP, CRP, and TNF-*α* (all *P* > 0.05), while after treatment, these indexes of both groups were improved, but the improvement in the obs group was more notable (*P* < 0.05). Additionally, the hospitalization time, treatment expense, readmission rate one year after discharge, and incidence of adverse events in the obs group were notably lower (all *P* < 0.05).

**Conclusion:**

For patients with both AMI and AHF, Entresto can contribute to strong amelioration of their clinical symptoms and prognosis and ventricular reverse-remodeling, with a high safety, so it is worthy of clinical promotion.

## 1. Introduction

Acute heart failure (AHF) is a disease in which systolic and diastolic dysfunction of the heart due to a variety of reasons results in the disturbance of blood flow from the heart, resulting in venous blood stasis and arterial hypoperfusion [1, 2]. It is a chronic and progressive clinical syndrome induced by structural or functional cardiac abnormalities [3]. In developed countries, AHF has become a substantial public health concern, affecting 2% of the adult population. Conventionally, AHF is mainly treated by ACEI or ARB, *β*-blocker, and aldosterone antagonist under synchronous diuretic and cardiotonic therapy. Current therapies are moderately effective at relieving the symptoms and signs of congestion by addressing the hemodynamic changes associated with AHF but have not demonstrated any benefit on long-term outcomes, presumably because they have limited effects on the underlying pathophysiology and fail to protect organs from damage in AHF [4]. At present, numerous studies confirmed that Entresto (sacubitril valsartan sodium) is more effective than enalapril in reducing the risk of death from AHF or cardiovascular disease in patients with stable AHF during hospitalization [5]. Entresto, mainly composed of sacubitril and valsartan, is the first angiotensin receptor enkephalinase inhibitor [6]. Sacubitril can promote sodium discharge, diuresis induction, blood vessel relaxation, and heart protection by enhancing the natriuretic peptide system, while valsartan can contribute to blood vessel relaxation, heart load reduction, and improvement of water-sodium retention by inhibiting renin-angiotensin-aldosterone and it further reduces both blood pressure and biomarkers of cardiovascular risk (troponin I and N‐terminal pro‐B‐type natriuretic peptide) [7, 8].

However, there is a paucity of studies reporting the application of Entresto in patients with both AMI and AHF. In this regard, this study we hypothesized that Entresto could yield beneficial results on the efficacy and ventricular remodeling (VR)-associated indexes and economic burden of the patients.

## 2. Materials and Methods

### 2.1. Participants

A total of 120 patients with AMI complicated with AHF (69 males and 51 females, with average (64.11 ± 5.29) years old) admitted to Tangshan Gongren Hospital between January 2017 and August 2019 were enrolled and randomly assigned to an observation group (obs group) and a control group (con group) at a ratio of 1 : 1. The obs group was treated with Entresto, while the con group with angiotensin-converting enzyme inhibitors (ACEI).

Inclusion criteria: patients meeting the diagnostic criteria of AMI combined with AHF, patients at II or III Killip classification, patients undergoing revascularization, patients with NT-proBNP ≥ 600 pg/ml, and those with an estimated survival ≥1 year. Exclusion criteria: patients with other severe comorbid systemic diseases that compromise the efficacy, patients with comorbid cardiac, liver or kidney dysfunction, patients with serious immune dysfunction, patients with paropsia, and those infected with bacteria, viruses or other pathogenic bacteria. All patients were informed of the study prior to signing informed consent, and the experiment was approved by the Ethics Committee of Tangshan Gongren Hospital (approval no. 71–141) and was in line with the *Declaration of Helsinki*.

### 2.2. Treatment Methods

All patients were given drugs when their hemodynamics was stable after admission. Those in the con group were treated with ACEI. Specifically, each patient was given 2.5 ml ACEI once a day initially, and then the dose was adjusted to an optimal one according to blood pressure and tolerance. Patients in the obs group were treated with Entresto. In essence, each patient was given 25 mg of Entresto twice a day initially, and then the dose was increased by 50 mg every 2–4 weeks until the maximum one of 200 mg (twice a day). The dose was adjusted according to the blood pressure and physical condition of the patients.

### 2.3. Outcome Measures

(1) The New York Heart Association classification (NYHA) was adopted to evaluate the clinical efficacy on the two groups after treatment [9]. Markedly effective: the NYHA of the patient reached class I or was improved by 2 classes; effective: the NYHA of the patient did not reach class I, but was improved by 1 class; ineffective: the NYHA of the patient had no change. The effective treatment rate = (the number of cases treated markedly effectively + the number of cases treated effectively)/the total number of cases × 100%. (2) The echocardiographic system was adopted to determine cardiac function-associated indexes: left ventricular end-systolic diameter (LVESd), left ventricular end-diastolic dimension (LVEDd), and left ventricular ejection fraction (LVEF) of the two groups, before treatment and after 1 month of treatment. (3) The patients' VR-associated indexes (interventricular septal thickness (IVST) and left ventricular mass index (LVMI)) were determined and compared before treatment and after 1 month of treatment. Additionally, NT-pro-BNP, CRP, and TNF-*α* of the two groups were tested and compared before and after treatment. (5) The hospitalization time, treatment expense, and readmission rate within one year after discharge in the two groups were recorded and compared. (6) Adverse events during follow-up among the two groups were recorded and compared, and the events included hypotension, hyperkalemia, elevated serum creatinine, angioedema, and cardiogenic shock.

### 2.4. Statistical Analyses

All data analyses were performed with SPSS20.0 (Bizinsight (Beijing) Information Technology Co. Ltd.), and the graphics visualization was conducted with GraphPad Prism 6. The enumeration data were verified by chi-square test, and the measurement data (mean ± standard deviation) were analysed via *t*-test. *P* < 0.05 was defined as a statistical difference.

## 3. Results

### 3.1. Comparison of General Data

The two groups were not notably different in sex, age, body mass index (BMI), smoking history, hypertension history, and diabetes mellitus history (*P* < 0.05) (Table 1).

### 3.2. Comparison of Efficacy

In the obs group, there were 36 patients of markedly effective, 22 of effective, and 2 of ineffective, while in the con group, the corresponding numbers were 23, 24, and 13, respectively. Overall, the obs group showed a notably higher total effective rate than the con group (96.67% vs. 78.33%; *P* < 0.05) (Table 2).

### 3.3. Comparison of Cardiac Function-Associated Indexes

Before treatment, there was no notable difference between the two groups in cardiac function-associated indexes (all *P* > 0.05); while after treatment, both groups had decreased LVEDs and LVEDd and increased LVEF (all *P* < 0.01), with the obs group having lower LVEDs and LVEDd and higher LVEF than the con group (*P* < 0.05) (Figure 1).

### 3.4. Comparison of VR-Associated Indexes

Before treatment, there was no notable difference between the two groups in VR-associated indexes (all *P* > 0.05), while after treatment, both groups showed decreased IVST and LVMI (*P* < 0.01), with significantly lower indexes in the obs group (both *P* < 0.05) (Figure 2).

### 3.5. Comparison of NT-proBNP, CRP, and TNF-*α*

Before treatment, there was no notable difference between the two groups in the levels of NT-proBNP, CRP, and TNF-*α* (all *P* > 0.05), while after treatment, the levels of them in both groups were improved (all *P* < 0.05), and the corresponding values in the obs group were notably lower (all *P* < 0.05) (Figure 3).

### 3.6. Comparison of Hospitalization Time, Treatment Expense, and Readmission Rate within One Year after Discharge

The hospitalization time, treatment expense, and readmission rate within one year after the discharge of the obs group were (5.97 ± 1.48) *d*, (24213.75 2576.44) Yuan, and 23.33%, respectively, while those of the con group were (9.55 ± 1.82) *d*, (49328.51 ± 3697.18) Yuan, and 53.33%, respectively. Overall the hospitalization time, treatment expense, and readmission rate within one year after the discharge of the obs group were greatly lower than those of the con group (all *P* < 0.05) (Table 3).

### 3.7. Comparison of Adverse Events

After treatment, the obs group had 2 patients with hypotension, 1 patient with hyperkalemia, 1 patient with elevated serum creatinine, 1 patient with angioedema, and 0 patients with cardiogenic shock, with an incidence of adverse events of 8.33%, while the con group had 4 patients with hypotension, 5 patients with hyperkalemia, 3 patients with elevated serum creatinine, 3 patients with angioedema, and 2 patients with cardiogenic shock, with an incidence of adverse events of 28.33%. The incidence of adverse events in the obs group was noticeably lower (*P* < 0.05) (Table 4).

## 4. Discussion

Over the past decades, the improvement of people's living standards and the change in lifestyle give rise to the incidence of cardiovascular disease and increase the incidence of AMI. AMI-induced AHF remains one of the leading causes of death associated with cardiovascular disease [10, 11]. For patients with AMI-induced AHF, aggressive measures to reduce cardiac load, relieve hemodynamics, and relieve symptoms are critical to improve prognosis [12].

In this study, we evaluated the efficacy and found that Entresto was more effective than enalapril. The possible explanation is that the Entresto formed in the sodium salt complex can effectively block angiotensin and inhibit enkephalinase to treat diseases, and can effectively improve the symptoms and cardiac function of patients, and delay the further development of the disease [13, 14]. In patients with AMI, myocardial remodeling involving various neurohumoral factors is a major cause of AHF [15]. Therefore, we also tested VR-related metrics in both groups and found that the obs group showed significantly better improvements in these metrics. According to reports [16, 17], Entresto has a dual-target regulation mechanism, and its mechanism of action is the same as that of enalapril. It can participate in natriuretic expansion, blood pressure reduction, myocardial remodeling reversal and cardiac function by inhibiting enkephalase and upregulating natriuretic peptide and bradykinin. The above results can confirm that Entresto can strongly relieve the clinical symptoms of patients and improve their cardiac function, thereby relieving the disease.

Among the biomarkers for assessing AHF, NT-proBNP, a natriuretic hormone, is considered an important laboratory test for the diagnosis of heart failure [18]. The increase of cardiac load will cause further stretch of ventricular myocytes, so that the compensatory synthesis of brain natriuretic peptides occurs in the blood circulation, and proteolytic enzymes are hydrolyzed into BNP and NT-proBNP in the blood circulation. NT-proBNP is specific to patients with cardiac insufficiency, with higher NT-proBNP levels indicating poorer cardiac function [19, 20]. As previously noted [21], inflammatory factors play a crucial role in promoting the pathogenesis of AHF, and their expression is bound up with disease severity and cardiac function of patients. Therefore, we also determined and compared NT-proBNP and serum inflammatory factors between the two groups before and after treatment, and the results showed that after treatment, NT-proBNP and serum inflammatory factors in both groups were improved, and the improvement in the obs group was more remarkable. The findings suggest that Entresto is effective in improving the inflammatory level of patients with AHF. For patients with AMI and AHF, long-term treatment and disease recurrence will not only bring great pain to the patients but also pose a heavy economic burden to the family [22]. Therefore, how to reduce the economic burden of patients while improving the efficacy of patients also needs to be considered. We found that the length of stay and the total cost of treatment were significantly lower in the obs group, suggesting that Entresto can not only shorten the length of hospital stay but also reduce the financial burden on patients. Importantly, we analysed the adverse events and readmission rates of patients in the two groups. The results showed that the incidence of adverse reactions and readmission rate of the obs group were notably lower, which suggests a good safety profile of Entresto.

In addition, acute heart failure can be classified as “heart palsy” and “palpitation” in traditional Chinese medicine. Traditional Chinese medicine believes that the heart dominates the blood vessels, and the spleen is easily affected by the deficiency of the heart and yang. If the yang qi of the heart and spleen are both deficient, the essence of water and grain cannot be metaplasticized, resulting in insufficient blood production. The normal heart function depends on the visible blood in the blood vessels, and insufficient blood production can cause the heart qi to be unable to promote blood flow, and finally form a vicious circle. Also, a previous study confirmed that Chinese herbal formula (50 g of semen ziziphi spinosae, 15 g of Rhizoma Angustifolia, 30 g of oyster, Bupleurum 25 g, 20 g of sun-cured ginseng, 20 g of *Rehmannia glutinosa*, 20 g of *Angelica*, 15 g of Radix Paeoniae Alba, 15 g of *Ligusticum wallichii*, and 10 g of cinnamon) has produced promising results. The possible explanation might be the followings: Semen ziziphi spinosae promotes fluid and soothes the nerves, Rhizoma nourishes Qi and promotes blood circulation, oyster calms the liver, sun-dried ginseng nourishes the heart and nourishes blood, *Rehmannia glutinosa* nourishes Yin and promotes body fluid, *Angelica sinensis* promotes blood and nourishes blood, and white peony root nourishes blood, *Ligusticum wallichii* removes blood stasis and relieves pain, while cinnamon promotes blood circulation and clears meridians. The combination of these medicines can play a role in nourishing heart Yin, invigorating heart Yang, and restoring blood vessels.

## 5. Conclusion

To sum up, for patients with both AMI and AHF, Entresto contributes immensely to melioration of clinical symptoms and prognosis, ventricular reverse-remodeling, rehabilitation, and economic burden ease, with a high safety profile. However, this study also has some limitations. First of all, since the number of cases we included is relatively small, it is necessary to further expand the sample size for further demonstration in the future. Second, we have not explored the specific mechanism of action of Entresto, so we should conduct further experiments in this regard to support our conclusions.

## Figures and Tables

**Figure 1:** Comparison of cardiac function-associated indexes between the two groups before and after treatment. (a) LVEDs. (b) LVEDd. (c) LVEF. ^*∗*^*P* < 0.05.

**Figure 2:** Comparison of ventricular remodeling-associated indexes between the two groups before and after treatment. (a) IVST. (b) LVMI.^*∗*^*P* < 0.05.

**Figure 3:** Comparison of NT-proBNP, CRP, and TNF-*α* between the two groups before and after treatment. (a) NT-proBNP. (b) CRP. (c) TNF-*α*. ^*∗*^*P* < 0.05.

**Table 1:** General data.

Factor	The observation group (*n* = 60)	The control group (*n* = 60)	*t*/*X*2	*P* value
Sex			0.367	0.580
Male	36 (60.00)	33 (55.00)		
Female	24 (40.00)	27 (45.00)		
Age (years)			0.302	0.583
≥64	31 (51.67)	34 (56.67)		
<64	29 (48.33)	26 (43.33)		
BMI (kg/m^2^)	22.85 ± 1.26	22.79 ± 1.31	0.226	0.799
Smoking history			0.136	0.713
Yes	27 (45.00)	25 (41.76)		
No	33 (55.00)	35 (51.47)		
Alcohol abuse history			0.391	0.532
Yes	14 (23.33)	17 (28.33)		
No	46 (76.67)	43 (71.67)		
Hypertension history			0.033	0.855
Yes	31 (51.67)	32 (53.33)		
No	29 (48.33)	28 (46.67)		
Diabetes mellitus history			0.367	0.580
Yes	33 (55.00)	36 (60.00)		
No	27 (45.00)	24 (40.00)		

**Table 2:** Evaluation of clinical efficacy of the two groups (*n*, (%)).

Efficacy	The observation group (*n* = 60)	The control group (*n* = 60)	*X*2	*P* value
Markedly effective	36 (60.00)	23 (38.33)	—	—
Effective	22 (36.67)	24 (40.00)	—	—
Ineffective	2 (3.33)	13 (21.67)	—	—
Total effective rate	58 (96.67)	47 (78.33)	9.219	0.003

**Table 3:** Comparison of hospitalization time, treatment expense, and readmission rate within one year after discharge.

	The observation group (*n* = 60)	The control group (*n* = 60)	T/*X*^2^	*P* value
Hospitalization time (days)	5.97 ± 1.48	9.55 ± 1.82	11.82	<0.001
Total treatment expense (Yuan)	24213.75 ± 2576.44	49328.51 ± 3697.18	43.17	
Readmission rate (*n* (%))	14 (23.33)	32 (53.33)	11.42	0.001

**Table 4:** Comparison of the incidence of adverse events between two groups (*n* (%)).

Adverse events	The observation group (*n* = 60)	The control group (*n* = 60)	*X* ^2^	*P* value
Hypotension	2 (3.33)	4 (6.67)	—	—
Hyperkalemia	1 (1.67)	5 (8.33)		
Elevated serum creatinine	1 (1.67)	3 (5.00)	—	—
Angioedema	1 (1.67)	3 (5.00)	—	—
Cardiogenic shock	0 (5.77)	2 (3.33)	—	—
Incidence of adverse events	5 (8.33)	17 (28.33)	8.015	0.005

## Data Availability

All the data generated or analysed during this study are included in this published article.
